# Construction of Diagnosis Model of Moyamoya Disease Based on Convolution Neural Network Algorithm

**DOI:** 10.1155/2022/4007925

**Published:** 2022-07-25

**Authors:** Xiangcheng Hao, Li Xu, Yin Liu, Cheng Luo, Yiming Yin, Xiao Chen, Xiaoyang Tao

**Affiliations:** Department of Neurosurgery, The Affiliated Suzhou Hospital of Nanjing Medical University, Suzhou 215000, China

## Abstract

**Objective:**

The convolutional neural network (CNN) was used to improve the accuracy of digital subtraction angiography (DSA) in diagnosing moyamoya disease (MMD), providing a new method for clinical diagnosis of MMD.

**Methods:**

A total of 40 diagnosed with MMD by DSA in the neurosurgery department of our hospital were included. At the same time, 40 age-matched and sex-matched patients were selected as the control group. The 80 included patients were divided into training set (*n* = 56) and validation set (*n* = 24). The DSA image was preprocessed, and the CNN was used to extract features from the preprocessed image. The precision and accuracy of the preprocessed image results were evaluated.

**Results:**

There was no significant difference in baseline data between the training set and validation set (*P* > 0.05). The precision and accuracy of the images before processing were 79.68% and 81.45%, respectively. After image processing, the precision and accuracy of the model are 96.38% and 97.59%, respectively. The area under the curve of the CNN algorithm model was 0.813 (95% CI: 0.718-0.826).

**Conclusion:**

This diagnostic method based on CNN performs well in MMD detection.

## 1. Introduction

Moyamoya disease (MMD) is a cerebrovascular disease characterized by chronic progressive stenosis or occlusion of the distal ends of bilateral internal carotid arteries followed by an abnormal vascular network at the base of the skull [1]. In the digital subtraction angiography (DSA), the compensatory vascular network showed a “smog” appearance, so it is called “MMD” [2]. MMD is most common in Asian countries such as Japan and China and affects women between the ages of 5 years and 40 years [3, 4]. MMD mainly presented with unilateral or bilateral stenosis or occlusion of the distal internal carotid artery, middle cerebral artery, and proximal anterior cerebral artery, accompanied by the formation of smoky and small vessels at the base of the brain and pia meningeal [5]. MMD includes ischemic and hemorrhagic blood types. In general, ischemic MMD is predominant in children and adults, and cerebral hemorrhage mainly occurs in adults. The mortality rate of hemorrhagic MMD is higher than that of ischemic MMD [6].

With the continuous development of medical technology, the commonly used diagnostic techniques of MMD mainly include magnetic resonance angiography (MRA), computed tomography angiography (CTA), and DSA [7]. The DSA is the gold standard for diagnosing MMD with high time and density resolution [8]. DSA imaging can not only clearly see the stenosis degree and the formation of smog-like vessels at the bifurcation of the internal carotid artery but also clarify the location and nature of vascular lesions, the establishment of collateral circulation, and the situation of extracranial vessels to intracranial compensation [9, 10].

DSA is a kind of angiographic video, which can provide richer vascular information, and MMD detection can be more effective on DSA [11]. With the development of biomedical engineering and artificial intelligence, deep learning has been widely used in medical diagnosis and treatment [12–14]. In this study, the diagnostic model of MMD was constructed based on the preprocessing DSA images by a convolution neural network (CNN), and its diagnostic value was discussed.

## 2. Materials and Methods

### 2.1. General Information

A total of 40 diagnosed with MMD by DSA from January 2016 to June 2018 in the neurosurgery department of our hospital were included in this study. The age ranged from 2.5 to 69 years, with a mean of 38 ± 3.9 years. Clinical symptoms include motor or sensory dysfunction, cognitive dysfunction, headache, involuntary movement, visual impairment, and transient ischemic attack. Postoperative follow-up was 6-39 months, with a median of 13 months. At the same time, 40 age-matched and sex-matched patients were selected. These patients with unrelated ischemic cerebrovascular disease and all patients were screened in the outpatient department of our hospital.

Inclusion criteria were as follows: (1) the patients met the guidelines for the diagnosis and treatment of MMD in adults and were diagnosed with MMD by DSA imaging and CT perfusion imaging; (2) conform to the operation indications; and (3) informed consent signed by family members. Exclusion criteria were as follows: (1) autoimmune diseases; (2) complicated with meningitis; (3) complicated with a brain tumor; (4) head trauma; (5) recently received head radiation; and (6) operative contraindications.

### 2.2. Image Preprocessing

Because of the need to prevent overlearning in the deep learning method, the training and verification sets of images are preprocessed. The first step is to remove the noise. The Gaussian filter function removed mechanical noise, and an algorithm removed moving noise. The second step is image enhancement. After denoising, histogram equalization is processed to increase the contrast difference between pixels in the image. The third step is image normalization (Figure 1). The enhanced data is normalized to near “0” to improve the training efficiency.

### 2.3. Construction of Convolutional Neural Network Model

In this study, CNN was used as the classifier of preprocessed images. Compared with traditional manual feature extraction methods, CNN can extract not only obvious features from images but also extract higher-level abstract features [15]. It alternately carries out convolution and pooling and then outputs the obtained features through the full connection layer to complete classification [16]. For the spatial limitations of images, the 2D convolution layer and pooling layer in 2D-CNN can be used to filter these limitations. The Conv2D convolution layer is used to extract image features, and the MaxPooling2D layer is used to reduce features and parameters and speed up training. The output of the convolution layer cannot be directly connected to the dense layer, so the flatten layer is needed to flatten the data of the convolution layer. The fully connected layer is used to combine features to reduce the impact of feature locations on classification, and the dropout layer can reduce overfitting and speed up training.

The activation function defines the output of the convolution kernel in the model. The activation functions used in this study include the ReLU function and Softmax function. The ReLU activation function used in the 2D convolution layer and the fully connected layer before the last layer can be expressed as follows:

(1) $$\begin{array}{c} \text{ReLU}\left(x\right)=\max\left(0,x\right). \end{array}$$

The activation function used in the last fully connected layer is the Softmax function, which can compress an arbitrary *k*-dimensional vector containing real numbers into another *k*-dimensional real vector so that the range of each element is in the interval of (0,1), and the sum of all elements is “1.”

(2) $$\begin{array}{c} \sigma {\left(z\right)}_{j}=\frac{e^{x^{T}w_{j}}}{\sum_{k=1}^{K}e^{x^{T}w_{k}}}\;\left(j=1,\cdots ,k\right). \end{array}$$

This output represents the probability value, representing the probabilities that fall into each category.

The loss function in a neural network is used to measure the difference between model training sample output and model output in the training stage. The loss function requires an optimizer to get the minimum. There are many loss functions in neural networks, and the cross-entropy loss function is commonly used in deep learning.

(3) $$\begin{array}{c} C=-\underset{y}{\sum }\ln\left(a\right). \end{array}$$

In this formula, *y* represents the real value, and *a* represents the output value of the model.

To make the deep learning network better learn the features of class *V* and class *S*, the loss function with weight coefficient is proposed in this study.

(4) $$\begin{array}{c} C=-\underset{ay}{\sum }\ln\left(a\right). \end{array}$$

In this formula, *α* is the weight coefficient. The value of *α* is 1 when the type is *N* and 5 in other cases. The optimizer used in this study was Adam, and the initial learning rate was 0.001.

The CNN structure used in this study is shown in Figure 2. Conv2D_1 and Conv2D_2 each contain two convolution layers, and the length and width of each convolution window are 3. Conv2D_1 output space dimension is 64, Conv2D_2 output space dimension is 128, and the activation function is ReLU. Conv2D_3 contains three convolution layers, the size of the convolution window is 3 × 3, the dimension of the output space is 256, and the padding of the convolution layer is the same. The step size of the maximum pooling layer is 2 × 2. The dropout layer has a ratio of 0.5.

### 2.4. Training of the Model

Subsequently, we randomly divided the data set into a training set (*n* = 56) and a verification set (*n* = 24) in a 7 : 3 ratio. After preprocessing, the training set data is used to construct the prediction model of deep learning, and then, the model is trained by CNN. Validation set data verifies the validity of the model. Then, the predictive efficiency of the model is evaluated. The specific process is shown in Figure 3.

### 2.5. Evaluation of the Model

All DSA images were preprocessed. The preprocessed images were trained by 5-fold cross-validation. The precision and accuracy of the preprocessed image results were evaluated. In addition, the prediction efficiency of the model was evaluated through the curve segment of receiver operator characteristic (ROC). The bigger the area under the curve, the higher the prediction efficiency.

### 2.6. Statistical Analysis

The Mann-Whitney *U*-test and Fisher's exact probability test were used to compare the data between the training set and validation set. All statistical analyses were conducted using the SPSS version 22.0 software (IBM, Armonk, NY, USA), and *P* < 0.05 was considered statistically significant.

## 3. Results

### 3.1. Data Comparison of Data Sets

In the training set, there were 22 male patients and 34 female patients. The mean age of the patients was 34.4 years. There were 28 patients with MMD. In the validation set, there were 10 male and 14 female patients, with an average age of 33.7 years. There were 12 patients with MMD. There was no significant difference in baseline data between the two groups (*P* > 0.05) (Figure 4).

### 3.2. Results of Image Preprocessing

DSA images are preprocessed with the same method, and the preprocessed images are detected. We obtained the related parameters of DSA image results before and after CNN processing. The precision and accuracy of the images before processing are 79.68% and 81.45%, respectively. After image processing, the detection performance is significantly improved, and the precision and accuracy of the model are 96.38% and 97.59%, respectively. The specific results were shown in Table 1.

### 3.3. Evaluation of the Effectiveness of Prediction Models

The prediction efficiency of the model was evaluated through the curve segment of the ROC. The ROC curve was shown in Figure 5. The area under the curve (AUC) of the CNN algorithm model was 0.813 (95% CI: 0.718-0.826).

## 4. Discussion

MMD has been known more and more since it was named in 1957 years [17]. However, the etiology of MMD is still unknown, and many factors such as heredity, immune system disease, and infection may be related to the formation of MMD to some extent [18]. The disease has a higher incidence in East Asia, particularly in Japan and China than in the United States [19]. The incidence of MMD was higher in females than in males. The peak of onset in adults is around 40 years old. The main clinical manifestations of MMD patients are transient ischemic attack, hemiplegia, cranial nerve disorder, headache, and dizziness. Some patients may also have visual field defect, epilepsy, syncope, and other symptoms [18, 20].

With the progress of imaging, more and more detection methods appear, such as MRA, CTA, and DSA [7, 21, 22]. This study constructs the MMD detection model based on the deep learning of the CNN algorithm. Firstly, the DSA image is preprocessed to extract the temporal and spatial features of DSA. The CNN algorithm can fine-tune the pretrained network in a small data set to prevent it from overfitting [23]. In this study, CNN was used as the classifier of preprocessed images. Compared with traditional manual feature extraction methods, CNN can extract noticeable features from images and higher-level abstract features [24]. For the spatial limitations of images, the 2D convolution layer and pooling layer in 2D-CNN can be used to filter these limitations. The pretrained Inception-ResNetV2 network is used to extract spatial features of DSA to help prevent network overfitting [25].

In patients with MMD, the stenosis or occlusion of the internal carotid artery system easily leads to insufficient cerebral blood supply and hypoperfusion of brain tissue, resulting in cerebral infarction or ischemia [26]. Therefore, early diagnosis of MMD patients is essential. This study constructs MMD diagnostic model based on the CNN algorithm. Because of the need to prevent overlearning in the deep learning method, the training and verification sets of images are preprocessed. In this study, there was no significant difference in baseline data between the two data. The same method was used to detect the images before and after preprocessing. The precision and accuracy of the images before processing are 79.68% and 81.45%, respectively, after 5-fold and cross calculation. After image processing, the detection performance is significantly improved (96.38% and 97.59%, respectively). Compared with the pretreatment, the detection accuracy of the model is increased by 15%. This shows that the diagnosis model based on deep learning has a good practical effect.

In addition, the diagnostic efficacy of the model was evaluated. The AUC of the CNN algorithm model was 0.813 (95% CI: 0.718-0.826). The area under the ROC curve is the AUC value. The larger the AUC is, the better the classification performance of the classifier will be. Thus, the better the detection effect will be.

## 5. Conclusions

This study diagnosed MMD based on CNN and performs well in MMD detection. This method provides a reference for the diagnosis of MMD in neurosurgery. This study has several limitations. First of all, CNN cannot process timing information. In image preprocessing, only the central part is input to reduce the influence of the surrounding background area. This will result in insufficient input images. In addition, due to a large number of original DSA sequences, the sequence images we selected are not necessarily the best choice. Finally, the number of patients enrolled in this study was small and single centers.

## Figures and Tables

**Figure 1:** Flow chart of image preprocessing in MMD.

**Figure 2:** Structure diagram of convolutional neural network.

**Figure 3:** Flow chart of the model training.

**Figure 4:** Data comparison between the training set and validation set. The difference between the two sets was not statistically significant (*P* > 0.05).

**Figure 5:** ROC curve of CNN prediction model.

**Table 1:** Diagnostic efficiency before and after image preprocessing.

Diagnostic efficiency	Before	After
Precision	79.68%	96.38%
Accuracy	81.45%	97.59%

## Data Availability

All data analyzed during this study are available from the corresponding author on reasonable request.

## References

[1] Huang S., Guo Z. N., Shi M., Yang Y., Rao M. (2017). Etiology and pathogenesis of moyamoya disease: an update on disease prevalence. *International Journal of Stroke*.

[2] Espert R., Gadea M., Alino M., Oltra-Cucarella J., Perpina C. (2018). Moyamoya disease: clinical, neuroradiological, neuropsychological and genetic perspective. *Revista de Neurologia*.

[3] Giustini A. J., Stone S. A., Ramamoorthy C. (2020). Moyamoya disease in children and its anesthetic implications: a review. *Paediatric Anaesthesia*.

[4] Inayama Y., Kondoh E., Chigusa Y. (2019). Moyamoya disease in pregnancy: a 20-year single-center experience and literature review. *World Neurosurgery*.

[5] Fang Y. C., Wei L. F., Hu C. J., Tu Y. K. (2021). Pathological circulating factors in moyamoya disease. *International Journal of Molecular Sciences*.

[6] Li J., Jin M., Sun X. (2019). Imaging of moyamoya disease and moyamoya syndrome. *Journal of Computer Assisted Tomography*.

[7] Shi Z., Ma G., Zhang D. (2021). Haemodynamic analysis of adult patients with moyamoya disease: CT perfusion and DSA gradings. *Stroke and Vascular Neurology*.

[8] Tian B., Jiang Y., Kang Q. (2018). Comparative study of 4D CTA and DSA for vascular assessment in moyamoya disease. *Clinical Imaging*.

[9] Cheon J. E. (2015). Quantitative digital subtraction angiography in pediatric moyamoya disease. *Journal of Korean Neurosurgical Association*.

[10] Song P., Qin J., Lun H., Qiao P., Xie A., Li G. (2017). Magnetic resonance imaging (MRI) and digital subtraction angiography investigation of childhood moyamoya disease. *Journal of Child Neurology*.

[11] Ge P., Zhang Q., Ye X. (2020). Postoperative collateral formation after indirect bypass for hemorrhagic moyamoya disease. *BMC Neurology*.

[12] Chan H. P., Samala R. K., Hadjiiski L. M., Zhou C. (2020). Deep learning in medical image analysis. *Advances in Experimental Medicine and Biology*.

[13] Li T., Fong S., Wong K. K. L., Wu Y., Yang X.-S., Li X. (2020). Fusing wearable and remote sensing data streams by fast incremental learning with swarm decision table for human activity recognition. *Information Fusion*.

[14] Meng C., Yang D., Chen D. (2021). Cerebral aneurysm image segmentation based on multi-modal convolutional neural network. *Computer Methods and Programs in Biomedicine*.

[15] Liu J., Zhao H. (2021). Application of convolution neural network in medical image processing. *Technology and Health Care*.

[16] Feng J., Chen J., Sun Q. (2021). Convolutional neural network based on bandwise-independent convolution and hard thresholding for hyperspectral band selection. *IEEE Transactions on Cybernetics*.

[17] Kondo T. (2018). Moyamoya disease. *CMAJ*.

[18] Mikami T., Suzuki H., Komatsu K., Mikuni N. (2019). Influence of inflammatory disease on the pathophysiology of moyamoya disease and quasi-moyamoya disease. *Neurologia Medico-Chirurgica (Tokyo)*.

[19] Li N., Luo P., Li C. (2021). Analysis of related factors of radiation pneumonia caused by precise radiotherapy of esophageal cancer based on random forest algorithm. *Mathematical Biosciences and Engineering*.

[20] Oh W. O., Shim K. W., Yeom I., Park I. T., Heo Y. (2021). Features and diversity of symptoms of moyamoya disease in adolescents: a cluster analysis. *Journal of Advanced Nursing*.

[21] Miyakoshi A., Funaki T., Fushimi Y. (2019). Identification of the bleeding point in hemorrhagic moyamoya disease using fusion images of susceptibility-weighted imaging and time-of-flight MRA. *AJNR American Journal of Neuroradiology*.

[22] Suzuki H., Mikami T., Komatsu K. (2017). Assessment of the cortical artery using computed tomography angiography for bypass surgery in moyamoya disease. *Neurosurgical Review*.

[23] Liang Q. (2021). Application of convolution neural network (CNN) model combined with pyramid algorithm in aerobics action recognition. *Computational Intelligence and Neuroscience*.

[24] Zhu T., Luo W., Yu F. (2020). Convolution-and attention-based neural network for automated sleep stage classification. *International Journal of Environmental Research and Public Health*.

[25] Li S., He X., Zhang H., Guo H., He X. End-to-end bioluminescence tomography reconstruction based on convolution neural network scheme.

[26] Suzuki H., Mikami T., Kuribara T. (2017). Pathophysiological consideration of medullary streaks on FLAIR imaging in pediatric moyamoya disease. *Journal of Neurosurgery. Pediatrics*.

